# Development of a Gene Risk Signature for Patients of Pancreatic Cancer

**DOI:** 10.1155/2022/4136825

**Published:** 2022-01-07

**Authors:** Tao Liu, Long Chen, Guili Gao, Xing Liang, Junfeng Peng, Minghui Zheng, Judong Li, Yongqiang Ye, Chenghao Shao

**Affiliations:** ^1^Department of Pancreatic-biliary Surgery, Changzheng Hospital, Navy Medical University, Shanghai, China; ^2^Department of Hepatobiliary Surgery, Heze Municipal Hospital, No. 2888, Caozhou Road, Mudan District, Heze 274000, Shandong, China; ^3^Department of Gastrointestinal Surgery, Heze Municipal Hospital, No. 2888, Caozhou Road, Mudan District, Heze 274000, Shandong, China; ^4^Department of Cardiology, Heze Municipal Hospital, No. 2888, Caozhou Road, Mudan District, Heze 274000, Shandong, China

## Abstract

**Background:**

Pancreatic cancer is a highly malignant solid tumor with a high lethality rate, but there is a lack of clinical biomarkers that can assess patient prognosis to optimize treatment.

**Methods:**

Gene-expression datasets of pancreatic cancer tissues and normal pancreatic tissues were obtained from the GEO database, and differentially expressed genes analysis and WGCNA analysis were performed after merging and normalizing the datasets. Univariate Cox regression analysis and Lasso Cox regression analysis were used to screen the prognosis-related genes in the modules with the strongest association with pancreatic cancer and construct risk signatures. The performance of the risk signature was subsequently validated by Kaplan–Meier curves, receiver operating characteristic (ROC), and univariate and multivariate Cox analyses.

**Result:**

A three-gene risk signature containing CDKN2A, BRCA1, and UBL3 was established. Based on KM curves, ROC curves, and univariate and multivariate Cox regression analyses in the TRAIN cohort and TEST cohort, it was suggested that the three-gene risk signature had better performance in predicting overall survival.

**Conclusion:**

This study identifies a three-gene risk signature, constructs a nomogram that can be used to predict pancreatic cancer prognosis, and identifies pathways that may be associated with pancreatic cancer prognosis.

## 1. Introduction

Pancreatic cancer is a highly malignant solid tumor [1], and its incidence and mortality rates continue to increase [2]. The most common symptoms in patients with pancreatic cancer are abdominal pain, anorexia, fatigue, and weight loss [3]; pancreatic cancer lacks specific biomarkers [4], and the main serum markers commonly used today are carcinoembryonic antigen and carbohydrate antigen 19-9; however, their sensitivity is not ideal [3]. Surgery is the most important approach in the treatment of pancreatic cancer. Due to atypical symptoms and the lack of effective screening tools, many patients have progressed to an unresectable state at the time of diagnosis. With the development of research, radiotherapy, chemotherapy, targeted therapy, and immunotherapy have been applied in the clinical treatment of pancreatic cancer with some success. However, for individual patients, a model that can effectively predict prognosis is still needed to guide clinical selection of treatment. The development of high-throughput sequencing technology has made it possible to discover prognosis-related biomarkers.

Weighted gene co-expression network analysis (WGCNA) has been used to detect correlations between gene modules consisting of highly correlated gene clusters and specific clinical features [5] and has been widely used to identify gene modules associated with clinical features of various cancers. In the present study, we identified gene modules highly correlated with pancreatic cancer tissue by WGCNA. In addition to this, we further identified genes associated with prognosis by univariate Cox regression analysis and Lasso Cox regression analysis.

## 2. Materials and Methods

### 2.1. Gene Expression Dataset Collection and Processing

Download datasets related to pancreatic cancer gene expression from GEO [6] (https://www.ncbi.nlm.nih.gov/geo/). The selection criteria in this article are (1) pancreatic cancer samples and normal samples were obtained from human samples; (2) the training and validation datasets needed to contain survival data; (3) using microarray gene-expression technology or RNA-Seq technology. Datasets GSE15471 [7], GSE16515 [8], GSE28735 [9], and GSE57495 [10] were selected for differential analysis and weighted gene co-expression analysis datasets, in which the GSE28735 dataset containing survival data was used to construct the prognostic gene signature; GSE78229 [11] was selected as the external validation dataset. Using the “sva” package [12] of *R* package, the GSE15471, GSE16515, GSE28735, and GSE57495 datasets are merged and normalized.

### 2.2. Differentially Expressed Gene Analysis and Weighted Gene Co-Expression Analysis (WGCNA)

Identification of differentially expressed genes (DEGs) by “limma” [13] package in *R*, setting |log Fold change (logFC)| ≥ 1 and adjusted *p* < 0.05 as standard. And we used “ggplot2” package [14] and “pheatmap” package [15] to plot heatmap and volcano map of DEGs. GO and KEGG enrichment analysis of the differential genes is carried out by *R* package “clusterProfiler” [16] and “GOplot” [17].

GSE15471, GSE16515, GSE28735, and GSE57495 data were merged, and weighted gene co-expression analysis was used to identify co-expressed gene modules using the “WGCNA” package [5] of R. GO and KEGG analysis was then applied to the genes within the module with the highest correlation to tumorigenesis.

### 2.3. Construction of Risk Signature

The univariate Cox regression and Lasso regression analyses of genes within the module were performed by the “survival” package [18] and “glmnet” package [19] to screen for prognosis-related genes within the module and construct a risk signature. Kaplan–Meier analysis was used to examine the survival outcomes of the high-risk and low-risk groups, and the predictive power of the risk signature was assessed using the area under the curve (AUC) of the controlled operating characteristic (ROC) curve. Prognosis-related genes were subsequently calculated in relation to risk score.

### 2.4. Construction and Valuation of Nomogram

Evaluation of prognostic factors are important for stage, grade, and risk score in the GSE78229 dataset by univariate and multifactor cox regression analysis using the “forestplot” package [20] in R. Nomogram which was drawn through “rms” package [21] and “regplot” package [22] to examine the accuracy of the nomogram by measuring the performance of the nomogram by the C-index. Calibration curves at 1, 3, and 5 years survival. Diagonal lines are used as a reference for best prediction. The *R* package “timeROC” was used by graph receiver operating characteristic curves (ROC) to determine the prognostic performance of the gene signature and nomogram.

## 3. Results

### 3.1. Differentially Expressed Genes' (DEGs) Identification

The GSE15471, GSE16515, GSE28735, and GSE57495 datasets were merged and normalized by the *R* package “sva” [12]. Subsequent differentially expressed gene analysis using the “limma” package [13] identified 77 DEGs containing 52 upregulated and 25 downregulated genes. We next performed GO and KEGG enrichment analysis of differential genes and plotted the circles. The GO analysis (Figure 1(c)) of their biological process (BP) was mainly enriched in extracellular structure organization and extracellular matrix organization; the cellular component (CC) was mainly enriched in proteinaceous extracellular matrix and extracellular matrix; the molecular function (MF) was mainly involved in extracellular matrix structural constituent and platelet-derived growth factor binding. However, no pathways were enriched in KEGG analysis.

### 3.2. Weighted Gene Co-Expression Network Construction and Key Module Identification

Weighted gene co-expression networks of GSE15471, GSE16515, GSE28735, and GSE57495 were constructed by the “WGCNA” package in *R* (version 4.0). The samples were clustered, and the sample clustering tree was drawn after removing the outliers (Figure 2(a)). We chose *β* = 7 (*R*2 = 0.9) to construct the scale-free network (Figure 2(b)). Eight co-expression modules were finally identified (which contained a grey module composed of genes that could not be categorized) (Figures 2(c) and 2(d)). Next, module-clinical feature correlation heat maps were drawn to assess the correlation between modules and clinical features (tumor vs. normal). The brown module had the strongest correlation with tumor tissue (*r* = 0.53 and *p*=7*e* − 22). Therefore, the brown module was selected as the key module for further analysis.

### 3.3. Construction of a Multigene Signature

Univariate Cox regression analysis was performed on 166 genes within the brown module to screen 30 genes associated with survival at *p* < 0.05, followed by Lasso Cox regression analysis in GSE28735 to calculate risk scores for pancreatic cancer patients. Risk score = (CDKN2A × 0.672) + (BRCA1 × −0.142)+(UBL3 × −0.185).

Patients were divided into a high-risk group (*n* = 21) and a low-risk group (*n* = 21) according to the median risk score. There was a significant difference in overall survival (OS) between the high- and low-risk groups (*p*=1.385*e* − 02) (Figure 3(c)). The areas under the curve at 1, 2, and 3 years was 0.75, 0.893, and 0.733, respectively (Figure 3(d)). The prognostic and prognostic accuracy of the three-gene signature was subsequently validated using GSE78229 as a test cohort. There was also a significant difference in OS between the high-risk and low-risk groups in the test cohort (*p*=5.418*e* − 03) (Figure 3(e)), with areas under the curve at 1, 2, and 3 years of 0.773, 0.731, and 0.741, respectively (Figure 3(f)).

The performance of the risk signature was further evaluated by univariate (Figure 4(a)) and multivariate (Figure 4(b)) Cox regression analysis in the train and test cohort, respectively. The results showed that the risk score was significantly associated with OS. Multivariate cox regression analysis revealed that three-gene signatures were independent predictors of outcome in pancreatic cancer patients.

In addition, we created a prognostic nomogram to help physicians predict overall patient survival in the clinic (Figure 4(c)). The calibration curve (Figure 4(d)) of the nomogram and the area under the curve of ROC (Figure 4(e)) showed a good concordance between prediction and observation.

## 4. Discussion

Pancreatic cancer is highly malignant, lacks reliable early screening methods, and has a poor prognosis, with an expected 5-year survival rate of approximately 9% [1]. Therefore, there is an urgent need to find biomarkers that affect the prognosis of pancreatic cancer in clinical treatment, which will facilitate the assessment of patient prognosis and will help to improve the prognosis by tailoring the treatment to the individual patient.

Tumor development is the result of multigene interactions, and therefore, an increasing number of risk signatures are used to predict prognosis [23–26]. In this study, we proposed a three-gene (CDKN2A, BRCA1, and UBL3) risk signature by WGCNA and Lasso Cox regression analysis for predicting overall survival in pancreatic cancer patients, with statistically significant differences in overall survival between high-and low-risk groups in the train cohort and test cohort. We then evaluated the prognostic performance of risk signature with the AUC of ROC, and the results showed that the risk signature could predict overall survival of pancreatic cancer patients accurately. Subsequent univariate and multivariate Cox analyses showed that the risk score could predict prognosis as an independent prognostic factor. In addition, we combined clinical characteristics to construct nomogram that can be used in the clinic to guide personalized treatment.

Among the risk genes we identified, CDKN2A (cytoskeleton-associated protein 2-like) was significantly highly expressed in the high-risk group and positively correlated with risk score; BRCA1 (glutathione S-transferase Mu 5) and UBL3 (Ubiquitin-like 3) were significantly down regulated in the high-risk group and negatively correlated with the risk score. CDKN2A has been reported to promote lung adenocarcinoma invasion and is correlated with poor prognosis [27]. Monteverde et al. found that CDKN2A could promote nonsmall cell lung cancer (NSCLC) progression by regulating transcriptional elongation, and targeting CDKN2A could enhance therapeutic response in patients with NSCLC [28]. Li et al. also found that CDKN2A knockdown inhibited proliferation, migration, invasion, and epithelial mesenchymal transition in glioblastoma cells [29]. Bioinformatics studies have found that CDKN2A is also associated with breast cancer [30], prostate cancer [31], and colorectal cancer [32]. BRCA1 has been reported to play an oncogenic role in bladder cancer, with significantly lower expression levels in cancer tissues than in normal tissues, and overexpression of BRCA1 reduced cell proliferation, migration, and colony-forming ability [33]. In contrast, in bladder cancer, upregulation of BRCA1 was able to resist oxidative stress, thereby promoting bladder cancer cell growth [34]. Pitt et al. also found mutations in BRCA1 in thyroid cancer. In addition to this, bioinformatics studies have found that BRCA1 is also associated with ovarian [35], colorectal [36], and gastric [37] cancers. Consistent with our speculation, Zhao et al. found that, in NSCLC, UBL3 acts as a tumor suppressor gene to inhibit cancer cell proliferation [38].

GSEA analysis revealed differences in 2 key signaling pathways between high- and low-risk groups. Base excision repair (BER) removes endogenous DNA damages that occur at all times in human cells, and its defects are associated with tumorigenesis [39], but cancer cells are also able to tolerate oxidative stress through increased BER activity, and targeting BER can improve the efficacy of radio/chemotherapy [40]. Our results show that the BER pathway is enriched in the high-risk group, suggesting that the BER pathway is active in high-risk patients, possibly leading to shorter survival by affecting their sensitivity to clinical treatment. An increasing number of studies have found that abnormal metabolism affects patient prognosis [41, 42], and the enrichment of propanoate metabolism pathway in the low-risk group suggests that the risk signature may affect patient prognosis through tumor metabolism.

In summary, our study identified a 3-gene risk signature for predicting prognosis, and the value of this risk signature was validated in an external test cohort. By combining this risk signature with clinical tumor pathology staging, a visual nomogram was created to facilitate the prediction of survival outcomes. We further analyzed risk signature-related signaling pathways and risk genes' expression and survival analysis in a variety of cancers, providing a research direction for exploring prognosis-related genes in in vivo and in vitro experiments. We further analyzed risk signature-related signaling pathways and risk gene expression and survival analysis in a variety of cancers, providing a research direction for exploring prognosis-related genes in cytological and animal experiments.

## Figures and Tables

**Figure 1:** Differentially expressed genes' (DEGs) identification. Heat map (a) and volcano map (b) of gene-expression profiles of pancreatic cancer tissues and normal tissues after merge of four datasets, GSE15471, GSE16515, GSE28735, and GSE57495. Differentially expressed genes were screened using |logFC| ≥ 1 and adjusted using *p* < 0.05, with red representing upregulated genes and blue representing downregulated genes. (c) GO enrichment analysis of differentially expressed genes.

**Figure 2:** Weighted gene co-expression network construction and key module identification. (a) Cluster dendrogram of pancreatic cancer samples and normal samples. (b) According to the scale-free index and the mean connectivity to screen soft threshold. (c) The cluster dendrogram of co-expression network modules. (d) Relationships between module and trait.

**Figure 3:** Construction of a multigene signature. (a) Univariate Cox analysis of genes within the brown module, screening of prognosis-related genes, and forest mapping. (b) The Lasso coefficient profiles of prognosis-related genes. (c) The partial likelihood deviance is plotted against log (*λ*). Kaplan–Meier plot of overall survival of patients is in the high-risk and low-risk groups in the train cohort (d) and test cohort (f). ROC curves for three-gene signatures in train cohort (e) and test cohort (g).

**Figure 4:** Evaluation of the predictive value of three-gene signatures and the creation of nomogram. (a) Test cohort risk signature univariate. (b) Multivariate Cox regression analysis forest plot. (c) Nomogram. (d) Calibration plot. (e) ROC curve for test cohort.

## Data Availability

The analyzed datasets generated during the present study are available from the corresponding author upon reasonable request.
